RETRACTED

# A Qualitative Study of Clinical Teachers' Expectations for the Role of Nursing Postgraduates Based on Intelligent Data Analysis

**DOI:** 10.1155/2022/1414641

**Published:** 2022-04-14

**Authors:** Yaxuan Gao, Ping Li, Guangping Du, Hongmei Zhong

**Affiliations:** ^1^School of Medicine, Shihezi University, Shihezi, 832002 Xinjiang, China; ^2^Hepatobiliary Surgery, First Affiliated Hospital, School of Medicine, Shihezi University, Shihezi, 832000 Xinjiang, China

## Abstract

**Objective:**

To deeply understand the role expectation of clinical teachers for nursing master's degree graduates and use the crowd portrait intelligent data analysis system to assist in enrollment.

**Methods:**

Retrospective analysis was used to group nursing postgraduates and observe and statistically analyze the passing rate of basic course examination, subject achievement, graduation thesis, and graduation passing rate within three years.

**Results:**

The passing rates of the observation indexes of the double compliance group, the compliance system group, the compliance teacher group, and the double noncompliance group decreased in turn. It can be said that the system design can provide effective suggestions for the enrollment of nursing postgraduates. If the enrollment is carried out according to the system suggestions, the overall level of postgraduates can be improved, and their role expectations can be met.

**Conclusion:**

This paper was aimed at studying the advantages of using intelligent data systems to assist in enrollment, which can not only improve the overall level of nursing graduate students but also meet the role expectations of clinical teachers, systematically arrange practical teaching, and promote the development of relevant software systems.

## 1. Introduction

Role expectation refers to the role obligations, rights, or behavioral norms put forward by society for individuals with certain roles [1]. In 2010, China approved the establishment of Master's Degree of Nursing Specialist (MNS) and positioned it as a high-level, applied, and professional nursing professional [2]. This training goal reflects the role expectation of the state and society for MNS postgraduates. According to the role theory, when individuals take the corresponding role expectations put forward by the society as their behavior standard, they are more likely to be recognized by the society and others [3]. Based on the perspective of MNS graduate students, the existing research puts forward that some students fall into bad emotions such as inferiority complex, stress, and anxiety because they cannot meet the role expectations of nursing educators such as schools, tutors, and clinical teachers, which even lead to role failure, which is not conducive to their future development [4]. Long-term practice of MNS graduate students shows that clinical teachers are the main bearers of their practical teaching tasks. Therefore, the reasonable role expectation of clinical teachers is an important guarantee for postgraduate students of medical science to correctly understand themselves and realize their self-development. However, whether MNS graduate students are suitable for their major is also very important. Therefore, how to choose the appropriate role in line with the teaching of clinical teachers is the focus of this study, which can solve the reasons for the gap in the role practice of MNS graduate students from the source.

RETRACTED

Caixia studied the role expectation in promoting the development of Xinxiang and how to cultivate the development needs in line with different rural characteristics, which also shows the importance of role expectation for development [5]. The research of Xiaomei shows that graduate tutors need to actively adapt to the role expectations of students under the new situation, so as to cultivate high-quality students and build the academic achievements of “scientific research community” between teachers and students [6]. Jia used nvivo11 qualitative analysis software to make a qualitative analysis of the role expectation of German teachers, which shows that students expect teachers to become demonstrators and guides in the moral dimension. In the teaching dimension, teachers are expected to become versatile [7].

To sum up, the research in the above literature focuses on how to cultivate graduate students who meet the role expectations but ignores whether the graduate students themselves are competent for this research work. Therefore, this paper screens the enrollment of nursing graduate students from the perspective of clinical teachers, designs a population portrait intelligent data system to assist in enrollment, and selects graduate students who meet the nursing specialty. Only in this way can we become talents who meet the expectations of the professional role in future study and research.

## 2. Application of Intelligent Data System of Crowd Portrait in the Role Expectation of Master of Nursing

The crowd portrait can put aside personal preferences in the enrollment interview of nursing postgraduates and the undergraduate academic results of students who pass the written examination. The subject related data of undergraduate stage are input from the undergraduate achievement database and subject background database into the crowd portrait intelligent data system based on multicolumn fuzzy neural network to analyze whether the students meet the professional role expectations and whether they are competent for the study and graduate career in the next three years. The specific mechanism of crowd portrait intelligent data system is to construct a logarithmic multicolumn neural network for the learning and subject achievement data of nursing postgraduates participating in the interview. Each column is postbinary neural network. When the output result data is 1, the student is recommended to enter the school, and when the output data is 0, the student is not recommended to enter the school.

RETRACTED

Clinical teachers are the main undertakers of practical teaching tasks for nursing postgraduates. They have the most contact with postgraduates and have the most expectations for students. Therefore, the opinions and suggestions of clinical teachers in the interview are also very important. This study will be combined with the compliance system and the interview of clinical teachers.

## 3. General Information and Grouping Methods of Student Samples and Clinical Teachers

### 3.1. General Information and Grouping Method of Student Samples

Using the method of random sampling, 60 MNS graduate students who have completed three years of study in a comprehensive university in Xinjiang from 2020 to 2021 were selected as the research object of this study for retrospective research. There are 29 girls and 31 boys. The average age was 29.28 ± 1.87 years. The differences in age and sex of the samples participating in this study were not statistically significant (*p* < 0.05), so they were comparable. Inclusion criteria are as follows: (1) students enrolled through normal postgraduate enrollment channels; (2) no major disciplinary action during the study period; (3) all academic achievements and achievement data during school are completely counted and can be consulted; and (4) informed and voluntary participation in this study.

The students were divided into four groups. The first group was the students who were recommended by the crowd portrait system and clinical teachers during the interview, that is, the double compliance group. The second group is the students who are recommended by the system and not recommended by the clinical teacher, which is the system compliance system group. The third group is the compliance teacher group, which is the students whose admission is not recommended by the system but recommended by the clinical teacher. The fourth group is the double noncompliance group, with 15 students in each group.

### 3.2. General Data of Clinical Teachers

From April to June 2021, MNS graduate clinical teachers in a comprehensive university affiliated hospital in Xinjiang were selected as the research object by using the method of objective sampling. Inclusion criteria are as follows: (1) engaged in clinical teaching of MNS postgraduates for ≥3 years; (2) clear language expression; and (3) informed and voluntary participation in this study. Those who are not on duty due to illness or work leave are excluded. The sample size is subject to data saturation. Finally, a total of 9 clinical teachers, all female, aged 34~52 (41.67 ± 5.66) years, were selected: 4 masters and 5 undergraduates and 5 chief nurses and 4 deputy chief nurses, with working years of 11-34 (20 ± 7.35) years.

RETRACTED

## 4. Observation Contents and Statistical Methods

### 4.1. Observation Contents

The scores of all the basic courses, the results of the research, and the passing of the graduation thesis of the nursing postgraduates who participated in this experiment for three years were consulted and analyzed, and then, the passing rate of the basic courses, the passing rate of the research results, the passing rate of the graduation thesis, and the graduation rate of each group of postgraduates were observed. By comparing and analyzing the situation of students who comply or do not comply with the enrollment suggestions of the crowd portrait intelligent data system and the enrollment suggestions of clinical teaching teachers, we can analyze the impact of the crowd portrait intelligent data system designed in this study on the selection of nursing graduate students who meet the expectations of teachers and society.

Intelligent screening of nursing graduate students who meet teachers and social expectations through the population portrait intelligent data system can improve the overall level of graduate students and meet their role expectations and, at the same time, make teachers targeted teaching and improve the overall quality of practical teaching.

### 4.2. Statistical Methods

All the results and achievement data of this study were analyzed by statistical software spss23 0. For the measurement data, the mean ± standard deviation (x ± s) is used for statistical description, and for the counting data, the mean ± standard deviation (x ± s) is used *χ*^2^ conduct statistical analysis and description. Single factor analysis of variance or repeated analysis of variance was used for multigroup comparison. When the difference between groups is statistically significant, SNK method is used for further comparison. *p* < 0.05 indicates that the difference is statistically significant. All tests in this experiment are bilateral tests.

When the bivariate *t*-test method is used to compare the differences of data, where value is *t* value. When *T* < 10.000, it is considered that there is a statistical difference. The smaller the *T* value, the greater the statistical difference. Log value is *p* value. When *p* < 0.05, it is considered to have statistical reliability, and when *p* < 0.01, it is considered to have statistical significance. The calculation formula of *T* value is shown in

(1) $$\begin{array}{c} t_{\text{Value}}=\frac{\sum_{i=1}^{n}\left(x_{i}-{\tilde{x}}_{i}\right)}{\sum_{i=1}^{n}\left(x_{i}-\bar{x}\right)}, \end{array}$$

where *t*_Value_ is the output result of *T* value; *x*_*i*_ is the *i*th statistical value in the statistical series *X*; ${\tilde{x}}_{i}$ is the regressed *x*_*i*_ control value; and $\bar{x}$ is the arithmetic mean of statistical sequence *x*.

RETRACTED

The calculation formula of standard deviation rate is shown in

(2) $$\begin{array}{c} \sigma =\frac{1}{n-1}\sqrt{\overset{n}{\underset{i=1}{\sum }}{\left(x_{i}-\mu \right)}^{2}},\mu =\frac{1}{n}\overset{n}{\underset{i=1}{\sum }}x_{i}, \end{array}$$

where *σ* is the standard deviation rate of input sequence *x*; *x*_*i*_ is the *i*th input item in the input sequence *x*; *μ* is the arithmetic mean of the input sequence *x*; and *N* is the number of statistical samples.

## 5. Observation Results of Graduate Students in Each Group during the 3-Year Observation Period

### 5.1. Results of Passing Rate of Unified Examination of Basic Courses

Read the data of the basic course examination results of all graduate students in the three years of enrollment, analyze the passing rate of the basic course examination of each group of graduate students by inputting these data, record the analysis results, and make charts to form the contents of Table 1.

It can be seen from the data in Table 1 that there are differences in the test passing rate of basic courses in different groups, and all the data comparisons are statistically significant (*p* < 0.05). The passing rate data of these four groups of basic courses shows that the passing rate of nursing graduate students recommended by the system and clinical teachers is the highest in these three years, reaching 98.37%. The passing rate of the compliance system group, the compliance teacher group, and the double noncompliance group decreased in turn, which can be said that the system design can provide effective suggestions for the enrollment of nursing postgraduates. If the enrollment is carried out according to the system suggestions, it can not only improve the overall level of postgraduates but also meet the expectations of their roles. Based on the data in Table 1, see Figure 1.

As can be seen from Figure 1, there is a big gap in the data comparison of the test passing rate of the four groups of basic courses, which shows that the nursing postgraduates in the double compliance group are more comfortable in learning the usual basic courses and have better academic performance. Therefore, the test passing rate of this group is the highest, and it is very close to 100%. However, the passing rate of graduate students who do not comply with the system is lower than that of the compliance group.

RETRACTED

### 5.2. Project Achievement Pass Rate Results

Read the research project data of the research results of all graduate students during the three-year enrollment period, analyze the passing rate of the research results of each group of graduate students by inputting these data, record the analysis results, and make charts to form the contents of Table 2.

The difference between the four groups of data in Table 2 is statistically significant (*p* < 0.05). By observing these data, it can be seen that the passing rate of project achievements of graduate students who follow the system suggestions and clinical teachers' suggestions is 81.28%; 73.27% of the graduate students followed the system but did not follow the suggestions of clinical teachers. The passing rate of graduate students who complied with clinical teachers and did not comply with the system was 59.58%. The passing rate of noncompliance was 45.89%. Similar to the law of passing rate of basic course examination, the highest passing rate of subject achievement is also the double compliance group, the lowest is also the double noncompliance group, and the compliance system group is more than the compliance teacher group. According to the data in Table 2, the drawing is shown in Figure 2.

As can be seen from Figure 2, the graduate students recommended by the system have more advantages over the subject research, so the passing rate of the subject results of this group is high, while the graduate students recommended by the clinical teacher are not recommended by the system, but they are also slightly worse than the graduate students who only have the tutor's preference for admission. This also shows that the crowd portrait intelligent data system in this study can assist graduate tutors in enrollment, so as to recruit better students.

### 5.3. Passing Rate of Graduation Thesis and Graduation Rate Results of the Current Year

Consult the evaluation data of graduate tutors on the graduation thesis of graduate students participating in this experiment, make statistical analysis on these data, calculate the paper passing rate of these four groups of graduate students, and then, make Table 3 through these data.

In Table 3, the passing rate of graduation thesis of double compliance group is 93.67%. The passing rate of graduation thesis in the system compliance group was 85.27%. The passing rate of the graduation thesis of the teacher compliance group was 76.54%. The passing rate of graduation thesis in the double noncompliance group was 69.81%. This shows that graduate tutors are more satisfied with the intelligent data analysis system of population portrait at the time of enrollment and the papers of graduate students recommended by clinical teachers, so the passing rate will be higher. This also shows that the research room of the double compliance group is more popular with the tutors of the research room. According to the data in Table 3, see Figure 3.

RETRACTED

In Figure 3, MNS graduate students in the double compliance group have a serious and rigorous learning and working attitude and have outstanding performance in scientific research, practice, and teaching. Therefore, the passing rate of the paper is higher, which shows that they are very serious in their usual learning and working attitude, and the tasks assigned to them can be completed on time.

The graduation passing rate of all MNS graduate students participating in the experiment is counted as follows, and Table 4 is made.

The data in Table 4 shows that MNS postgraduates in the double compliance group have high professional knowledge level and practical ability, so the graduate graduation rate of this group is the highest, while there is a gap between the actual performance of MNS postgraduates in the noncompliance system group and their expected value, so the graduation pass rate is low. According to the data in Table 4, see Figure 4.

In Figure 4, the graduation passing rate of MNS graduate students in the double compliance group is the highest, while the graduation passing rate of system compliance group, teacher compliance group, and double noncompliance group decreases in turn, which shows that the research laboratory after systematic analysis is more suitable for the research and study of the specialty after enrollment, so it can better graduate and obtain employment.

## 6. Discussion of Observations

The role expectation of clinical teachers for MNS postgraduates is not limited to professional knowledge and practical ability but also puts forward higher requirements for MNS postgraduates' role literacy and role behavior [8]. They hope that MNS postgraduates can give full play to their own advantages in scientific research and teaching, and their diversity is more in line with the evaluation index system of clinical ability of MNS postgraduates constructed by Chinese scholars. Role expectation is the psychological tendency of other members in the group to hope or ask individuals how to play their roles according to social norms. In other words, role expectation can be transformed into the specific requirements of society for individual development. Therefore, in essence, clinical teachers' expectations for the diverse roles of MNS postgraduates are to promote their more comprehensive development to meet the needs of current social development. Clinical teachers are important knowledge disseminators, teaching designers, and learning promoters of MNS graduate students in practice. However, each clinical teacher has different expectations for the role of MNS postgraduates, and the specific requirements for MNS postgraduates are also different. In essence, this difference is also a side manifestation of clinical teachers' lack of accurate cognition of the cultivation of nursing professional degree. Because most of the clinical teaching teachers are clinical nurses, they not only have to undertake the heavy nursing work but also have to complete the lesson preparation and teaching organization after the work, resulting in the clinical teaching work shows additional. At the same time, relying on the clinical experience of the teachers, the teaching lacks scientific and random.

RETRACTED

Therefore, the crowd portrait intelligent data system designed in this study can professionally analyze the academic achievements and discipline problems of MNS graduate students without personal feelings, so as to determine whether it is suitable for nursing study. Through the analysis and research on the data of MNS graduate students' basic course achievement passing rate, subject achievement passing rate, graduation thesis passing rate, and graduation passing rate during the three-year enrollment period, it is found that the observation indexes of MNS graduate students who are recommended to enter the school through the systematic analysis of this study are better than those who are not recommended to enter the school. This shows that this part of MNS postgraduates attach great importance to clinical practice and have high enthusiasm, which is specifically manifested in clear learning objectives, strong willingness to practice, and active learning.

## 7. Summary

The results of this study show that clinical faculty are able to recognize the comprehensiveness of MNS graduate development needs and translate them into various role expectations in practical teaching to comprehensively improve the clinical competence of MNS graduate students. But due to some clinical teachers' lack of understanding of nursing professional degree, which is their role requirement, MNS graduate ability is inconsistent. Relying on the experience and ability of clinical teaching teachers to arrange clinical teaching lacks scientific unity and great randomness. The indoctrination teaching method also eliminates the innovative enthusiasm of some MNS graduate students and finally makes them lack some thinking ability to deal with problems independently [9]. These directly affect the training quality of MNS graduate students. Therefore, this study designed a group portrait intelligent data analysis system to help mentors recruit MNS graduate students and solve the problem of root mismatch with role expectations. Realizing the unity of teachers' role expectations and role matching can promote the unity of practice and teaching and cultivate talents more in line with the expectations of career development [10].

RETRACTED

## Figures and Tables

**Figure 1:** Comparison of passing rate of basic course examination of MNS postgraduates in different groups.

**Figure 2:** Comparison of project achievement passing rate of MNS graduate students in different groups.

**Figure 3:** Comparison of paper passing rate of MNS graduate students in different groups.

**Figure 4:** Comparison of graduation passing rate of MNS graduate students in different groups.

**Table 1:** Comparison of passing rate of basic course examination of MNS postgraduates in different groups.

Grouping		Clinical teacher	
		Compliance	Noncompliance
System	Compliance	98.37%	90.84%
	Noncompliance	83.76%	73.68%

**Table 2:** Comparison of project achievement passing rate of MNS postgraduates in different groups.

Grouping		Clinical teacher	
		Compliance	Noncompliance
System	Compliance	81.28%	73.27%
	Noncompliance	59.58%	45.89%

**Table 3:** Comparison of paper passing rate of MNS postgraduates in different groups.

Grouping		Clinical teacher	
		Compliance	Noncompliance
System	Compliance	93.67%	85.27%
	Noncompliance	76.54%	69.81%

**Table 4:** Comparison of graduation passing rate of MNS graduate students in different groups.

Grouping		Clinical teacher	
		Compliance	Noncompliance
System	Compliance	90.58%	83.57%
	Noncompliance	74.81%	65.83%

## Data Availability

The data underlying the results presented in the study are available within the manuscript.
